The article "LSGDM with Biogeography-Based Optimization (BBO) Model for Healthcare Applications" was published in 2022. Journal: J Healthc Eng.

# LSGDM with Biogeography-Based Optimization (BBO) Model for Healthcare Applications

**DOI:** 10.1155/2022/2170839

**Published:** 2022-04-30

**Authors:** A. Harshavardhan, Prasanthi Boyapati, S. Neelakandan, Alhassan Alolo Abdul-Rasheed Akeji, Aditya Kumar Singh Pundir, Ranjan Walia

**Affiliations:** ^1^Department of CSE, VNR Vignana Jyothi Institute of Engineering and Technology, Hyderabad, India; ^2^Department of CSE, R.V.R & J.C College of Engineering, Guntur, India; ^3^Department of CSE, R.M.K Engineering College, Chennai, India; ^4^Department of Marketing and Corporate Strategy, Tamale Technical University, Tamale, Ghana; ^5^Department of ECE, Arya College of Engineering and Information Technology, Jaipur, India; ^6^Department of Electrical Engineering, Model Institute of Engineering and Technology, Jammu, India

## Abstract

Several studies aimed at improving healthcare management have shown that the importance of healthcare has grown in recent years. In the healthcare industry, effective decision-making requires multicriteria group decision-making. Simultaneously, big data analytics could be used to help with disease detection and healthcare delivery. Only a few previous studies on large-scale group decision-making (LSDGM) in the big data-driven healthcare Industry 4.0 have focused on this topic. The goal of this work is to improve healthcare management decision-making by developing a new MapReduce-based LSDGM model (MR-LSDGM) for the healthcare Industry 4.0 context. Clustering decision-makers (DM), modelling DM preferences, and classification are the three stages of the MR-LSDGM technique. Furthermore, the DMs are subdivided using a novel biogeography-based optimization (BBO) technique combined with fuzzy C-means (FCM). The subgroup preferences are then modelled using the two-tuple fuzzy linguistic representation (2TFLR) technique. The final classification method also includes a feature extractor based on long short-term memory (LSTM) and a classifier based on an ideal extreme learning machine (ELM). MapReduce is a data management platform used to handle massive amounts of data. A thorough set of experimental analyses is carried out, and the results are analysed using a variety of metrics.

## 1. Introduction

Recent technologies, such as big data, the internet of things (IoT), wearables, and so on, have a significant impact on society, healthcare organisations, and our daily lives. Big data plays an important role in obtaining the necessary data during the decision-making process. Big data is defined as a complex and massive volume of data derived from various sources and clinical data sets that provide critical information for patient treatment [1]. Furthermore, big data has the potential to improve healthcare operations through data-driven decision-making in the ambiguous environment of Industry 4.0. Big data analytics provide significant benefits for evaluating and assimilation of massive amounts of complex healthcare data. The medical system keeps track of the world's most pressing social and economic issues in order to find innovative solutions through technology and science. The Industry 4.0 model was first proposed in 2011, and it was initially referred to as the production or manufacturing process. While incorporating, medical services and Industry 4.0 are complementary methodologies. Furthermore, with the rise of big data and the widespread use of electronic healthcare records of patients in healthcare organisations, chasing solutions to population medical problems is no longer viable. Using big data for better decision-making, on the other hand, poses some healthcare challenges.

In recent years, group decision-making has received a lot of attention in various areas of healthcare organisations [2]. The more severe the challenge, the more complex it can withstand the loss caused by a decision-making error. As a result, many civil organisations and government departments, as well as managers and experts in various fields, would be involved in decision-making. Based on the preferences of decision-makers, LSGDM selects sufficient alternates from a group of possible alternates [3]. When the number of decision-makers (DM) increases, the standard group decision-making problem transforms into the LSGDM problem. LSGDM problem-solving methods typically consist of four phases: (i) the cluster standardised individual decision matrices, (ii) standardising original individual decision metrics, (iii) selecting the best alternatives, and (iv) aggregating the cluster decision metrics.

Based on the conventional decision-making method, the current study significantly innovates by incorporating four factors: distinct decision-makers' preference data expression, attribute weight determination method, large-scale group clustering method, and large group preference data aggregation method [4]. One of the most common fields of study is large-scale group preference data aggregation. Despite the fact that the number of studies deliberating big data is steadily increasing, applications of large-scale group decision-making procedures in the context of big data studies and medical Industry 4.0 remain rare. This work creates a new MapReduce-based LSDGM model (MR-LSDGM) for the Industry 4.0 environment to improve decision-making in healthcare management. With the rapid advancement of information technology, as exemplified by the Internet, decision support systems will evolve toward socialisation in the era of big data. This is because DMs from various areas can be invited to collaborate on difficult issues on a single network platform. Simultaneously, we can conduct online voting on a particular item and perform automated statistical analysis. Additionally, it may analyse and research multitemporal and group events, such as those on e-commerce websites and search engines, to provide critical data support for qualitative decision-making. It appears to be worthwhile to develop large-scale group support tools to aid in decision-making, given that the big data era may contain a variety of data sources, including social media, mobile devices, and websites. Several researchers have developed software implementations of LSGDM, including the WTALGDM for LSGDM on energy network dispatch optimization, MENTOR for visualizing opinion evolution, and a multiagent system model for assisting with CRP. Other application fields, such as healthcare and engineering, require the use of these tools. A large number of simulations are run to demonstrate the improved results of the MR-LSDGM technique, and the experimental findings are examined using several metrics.

## 2. Related Works

Li and Wei [5] created an LSGDM model for making medical management decisions. For describing the decision data, the HFLTS is used. For clustering the DM into many subgroups, a clustering technique based on the ideal point is presented. The DM preference is then combined with the PDEHFLTS model to retain the decision data. A subgroup weight method is proposed for calculating the ranking weight based on the subgroup size and the presented hesitant entropy of PDEHFLTS. For large-scale GDM problems, Li et al. [6] used a fuzzy cluster analysis to integrate heterogeneous data. Fuzzy cluster analysis is used to divide large groups into smaller ones, and F-statistics are used to calculate the number of clusters required. The original data is kept depending on the degree of similarity. A consensus-building process is then used among these smaller groups to reach a common understanding. While other groups could not agree, a feedback system was devised to update the smaller GDM matrix, and the TOPSIS model was used to select the best option.

Song and Yuan [7] proposed a new GDM method based on arithmetic programming and employing IMGFLPR. As a result, a consensus procedure based on IMGFLPR is developed, while dynamic adaptation of expert weights is considered. Finally, problems with emergency plan election are solved using the presented method, which demonstrates the effective outcome of GDM. Wan et al. [8], inspired by multiplayer game concepts, proposed a two-step optimization algorithm that first maximises individual fulfilment while minimizing group conflict. The provided approach effectively saves decision-making time when it comes to ensuring the quality of LSGDM.

Hsu et al. [9] identified eight potential developments for providing a proper approach to the medical industry. The modified Z-DEMATEL method is used to build the mutually important relationship and prioritises this trend. By optimising the classic fuzzy number and representing the assessment environments' confidence under uncertainty, the Z-number technique improves the consistency of expert evaluation. Liu et al. [10] developed an LGDA approach for managing dependency in HRA based on the interval two-tuple linguistic variable and cluster analysis model. In addition, an expanded Muirhead mean operator was developed to determine the amounts of reliance between the activities of consecutive operators. Finally, empirical medical dependency analysis is used to demonstrate the applicability and effectiveness of the presented LGDA model [11].

Du and Shan [12] proposed a dynamic intelligent integration suggestion approach for product ideas. They began by creating one-of-a-kind product concept assessment condition systems that included both output and input criteria. The following section describes a step for static data combination and data extraction. Later, the fundamental likelihood assignments function is used as a data extraction approach to accurately reflect and effectively capture the validity of experts' evaluations. Dursun et al. [13] proposed a fuzzy multicriteria GDM architecture based on the fuzzy integral and measure principle to evaluate the HCW treatment alternatives for Istanbul. In the case of the GDM problem, an expert consensus is required for the calculation method to be carried out correctly. The OWA operators are used in this work to aggregate DM opinions.

Pan et al. [14] concentrated on using dynamic programming to solve the large-scale GDM problem, in which the data is in the form of linguistic variables. Because the linguistic variable cannot be directly computed, the interval type-2 fuzzy set is used for encoding. The distinct similarity and distance models are then constructed concurrently in order to determine the relationship between the interval type-2 fuzzy set. Later, a dynamic programming approach based on clustering models was presented for clustering the DM from an overall perspective. Gao et al. [15] created a novel paradigm for selecting an appropriate physician in the index system that balances the 2D calculation result. The researchers created questionaries and conducted field research to bring the given technique closer to the actual situation in China. They then calculated the best outcome for the best medical services provided by doctors [16].

## 3. The Proposed MR-LSDGM Technique

The MapReduce tool is used in this study to create a new MR-LSDGM approach for the healthcare industry. The MR-LSDGM approach includes BBO-FCM-based DM clustering, 2TFLR-based preference modelling, and LSTM-OELM-based classification procedures. The proposed MR-LSDGM model is depicted in its entirety in Figure 1. The MapReduce tool is used by the MR-LSDGM approach to managing massive amounts of data in the healthcare industry. The sections that follow provide a more detailed explanation of these processes [17].

### 3.1. MapReduce

The primary goal of the Map procedure is to compute the geometric distance between cluster centres and sampling point data. Read the data from Hadoop Distributed File Systems (HDFS) and use the stated (value, key) pair input formats as Map function input values, where “key” denotes the sampling point data ID numbers and “value” means the entire data sampling point and then read the maximal consumption. The minimal distance approach would evaluate the major cluster centre, compute Euclidean distances between other cluster centres using sample point data, and integrate the membership degree (MD) [18].

The primary goal of Reduce functions, on the other hand, is to obtain a large number of Map function outputs. To begin, obtain the key values pair from the Map functions, where “key” represents the cluster centres and “value” represents the sampling point data equivalent to the cluster centres. The data sample from a number of distinct cluster centres is then merged, and a new cluster centre is evaluated. Finally, it is determined whether the geometric distance between the novel and equivalent cluster centres exceeds a predetermined threshold or whether the number of iterations exceeds that threshold.

Despite outperforming traditional hard clustering algorithms in terms of clustering effects, fuzzy clustering algorithms have a few drawbacks. The current clustering algorithms are extremely sensitive to early clustering centres. Because the algorithms use the concept of gradual iteration, the objective functions are continuously reduced during the iteration. As a result, when the *c* clustering centre is arbitrarily chosen in each sample data set at first, the geometric distance that would produce the last clustering results for falling to the current optimum solution is smaller. To avoid situations in which the geometric distance between the arbitrarily chosen cluster centre is smaller, the minimum and maximum distance methods were used to determine the early cluster centre in this study.

### 3.2. Design of BBO-FCM Technique

In the beginning, the BBO-FCM approach is used to divide the DMs into subgroups. Every feature vector with a coefficient between [0, 1] belongs to one of the FCM clusters. Finally, the algorithm labels all of the data points (feature vectors) based on the maximum coefficient of these data points across all clusters. By minimizing the following equation, the cluster centre and fuzzy membership matrix are calculated.

(1) $$\begin{array}{c} \sum_{g=1}^{c}u_{i,j}=1, \end{array}$$

where *u* represents the sum of data; *c* indicates the quantity of clusters; *u*_*g*,*j*_ signifies the fuzzy association of *j*th point to *i*th clusters; *d*_*g*,*j*_ means the cluster centres and data point *l* ∈ (1, *∞*), a fuzzy weight factor that determines the quantity of fuzziness produced as a result In most cases, and *l* = 2 is chosen (it can be stated that this value of *m* does not generate optimum solutions for each problem).

Because of the constraints in (1), all points must completely allocate their memberships to each cluster [19]. The fuzzy weight centre of gravity of the data is used to define the cluster centre (centroid)X.

(2) $$\begin{array}{c} v_{j}=\;n\sum_{j=1}^{n}u_{i,j},x^{l}x_{j}. \end{array}$$

As *u*_*g*,*j*_ influences the calculation of the cluster centres *ν*_*i*_, data with more memberships would have a greater influence on the prototype position than data with fewer memberships. Because *u*(*g*, *j*) has an effect on the calculation of the cluster centres *v*_*i*_, it is necessary to consider it. The distance *d*_ is used in the fuzzy C-means technique (*g*, *j*). Clustering using fuzzy logic (sometimes referred to as soft clustering or soft k-means) allows each individual data point to be assigned to more than one cluster. For fuzzy *C*‐means approach, distance *d*_*g*,*j*_ is determined by

(3) $$\begin{array}{c} d_{g,j}u^{2}={\left\|x_{j}-v_{i}\right\|}^{2}. \end{array}$$

The cluster centre *v*_*i*_ represents the common value of that cluster, where the *u*_*g*,*j*_ components of the association matrix denote the range where the data point *x*_*j*_ is related to its model. The minimalization of divide function (1) would derive the following equation:

(4) $$\begin{array}{c} \frac{d_{g,j}}{d_{g^{j}}},x^{1/\left(l-1\right)}+u_{g,j}=\frac{1}{2}. \end{array}$$

Equation (4) is defined in an iterative manner as the distance *d*_*g*,*j*_ is based on membership *u*_*i*,*k*_. The process to compute the FCM is given below:

- Opt for the number of cluster *c*, 2 ≤ *c* < *n*; select *m*, 1 ≤ *l* < *∞*.Initialize*U*^(0)^.
- Compute the cluster centre *ν*_*i*_ by (2).
- Compute the novel partition matrix *U*^(1)^ by (4).
- Relate *U*^(*j*)^ & *U*^(*j*+1)^. When the variations of the MD *u*_*k*,*i*_ computed by proper standards are smaller when compared to the provided threshold, end the process and return to step (2).

The BBO algorithm is used to define the optimal initial cluster centre of the FCM technique. The BBO has a population-based optimised technique that simulates the development and the balance of predator and prey in different ecosystems. According to research, the BBO produces better results than the other population-based techniques [20]. This technique utilises the BBO algorithm to select the optimal initial cluster centre to use for its initial cluster centre determination process. For each setting, the BBO uses an optimal population-based technique to simulate development and the balance between predators and prey. It has been discovered through research that the BBO generates superior results when compared to other population-based approaches. From one iteration to the next, a collection of solutions is retained, and all habitats send and receive inhabitants. The various habitats are determined by their immigration and emigration rates, which are probabilistically modified. An arbitrary number of habitats are occasionally mutated during all iterations. All of the solution parameters are now referred to as suitability index variables (SIV). Simon was the first to propose the concept of a biogeography-based optimization method. Using the scientific understanding of migration and the dispersion of species from one habitat to another, this method has been devised and tested. Each location has a habitat suitability index (HSI), which is based on the concepts of this algorithm and acts in a similar way to the fitness function in other population-centred algorithms. In addition, the suitability index variables refer to the independent factors that are used to determine the suitability index of a settlement (SIV).

The mathematical method of immigration (*λ*_*k*_) and emigration (*μ*_*k*_) is expressed as follows:

(5) $$\begin{array}{c} \lambda_{k}=I\left(1-\frac{S_{k}}{S_{\text{max}}}\right),\\ \mu_{k}=E\left(\frac{S_{k}}{S_{\text{max}}}\right), \end{array}$$

where *I* refers to the maximal rate of immigration, *E* defines the maximal rate of emigration, *S*_max_ implies the maximal number of habitats, and *S*_*k*_ represents the habitant count of *k*.

The following are the modifications to all habitats that improve the evaluation of BBO:

(6) $$\begin{array}{c} m\left(s\right)=m_{\text{max}}\times \left(1-\frac{P_{n}}{P_{\text{max}}}\right), \end{array}$$

where *m*_max_ represents the higher value of mutation determined as a user, *P*_max_ demonstrates the superior mutation probabilities of every habitat. and *P*_*n*_ refers to the mutation probabilities of *n*^th^ habitat that is given by

(7) $$\begin{array}{c} \overset{´}{P_{n}}=\left\{\begin{array}{cc} -\left(\lambda_{n}+\mu_{n}\right)P_{n}+\mu_{n+1}P_{n+1}, & n=0;\\ -\left(\lambda_{n}+\mu_{n}\right)P_{n}+\mu_{n+1}P_{n+1}+\lambda_{n-1}P_{n-1}, & 1\leq n\leq S_{\text{max}}-1=0;\\ -\left(\lambda_{n}+\mu_{n}\right)P_{n}+\lambda_{n-1}P_{n-1}, & n=S_{\text{max}}. \end{array}\right. \end{array}$$

At this point, $\begin{array}{c} \emptyset ⟶\left\{H^{n},HSI^{n}\right\}\\ I: \end{array}$ sets an ecosystem of habitat and calculates all equivalent HSIs, and Γ=(*n*, *m*, *λ*, *τ*, Ω, *M*) describes the function that switches from one optimised cycle to the next. The six tuples of elements are described, where *n* implies the number of habitats, *m* refers to the number of SIVs, *λ* represents the rate of immigration, *τ* demonstrates the rate of emigration, Ω refers to the migration function, and *M* indicates the mutation operator.

### 3.3. Modelling Preferences of DMs Using 2TLFR Technique

Once the DMs have been clustered, their perspectives can be defined and fused using the 2TLFR technique to retain as much decision information as possible. Decision-making in healthcare is based on dynamic conditions and ambiguous information, and most decision-makers prefer linguistic variables or fuzzy values over hard numbers. In the two-tuple linguistic depiction method, the data measured in the linguistic hierarchy term set could be unified with no data loss.

**Definition 1 .**

*S*={*s*_0_, *s*_1_,…, *s*_*g*_} represents a linguistic term set; *βϵ*[0, *g*] denotes the outcome of an aggregation index of a group of labels measured in *S*.(*s*_*γ*_, *α*) indicates linguistic two tuples; *s*_*γ*_*ϵS* and *αϵ*[−0.5, 0.5]; *s*_*γ*_ characterises the linguistic label of the data; and *α* means the mathematical value that expresses the values of the translation from the original results *β* to the nearest index label *γ* in *S*, namely, the symbolic translation.

The following function converts mathematical numbers and linguistic two tuples. They can convert mathematical values to linguistic two tuples using (9) [8].

(8) $$\begin{array}{c} \Delta :\left[0,g\right]⟶s\times , \end{array}$$

(9) $$\begin{array}{c} \Delta \left(\beta \right)=\left\{\begin{array}{cc} s_{\gamma }, & \gamma =\text{round}\left(\beta \right),\\ \alpha =\beta -r, & \alpha \in \left[-0.5,0.5\right]. \end{array}\right. \end{array}$$

Using the eq., they can convert a linguistic phrase to a real value (between 0 and *g*).

(10) $$\begin{array}{c} \Delta^{-1}:s\times \left[-0.5,0.5\right]⟶\left[0,g\right]\\ \Delta^{-1}\left(s_{\gamma },\alpha \right)=\gamma +\alpha =\beta \end{array}$$

To further unify the dimension, they could use the eq. to map the linguistic term between zero and one.

(11) $$\begin{array}{c} \Delta^{-1}:s\times \left[-0.5,0.5\right]⟶\left[0,1\right],\\ \Delta^{-1}\left(s_{\gamma },\alpha \right)=\frac{\gamma +\alpha }{g}. \end{array}$$

### 3.4. Automated Disease Classification Model

Finally, the disease classification process is divided into three stages: feature extraction using LSTM, classification using ELM, and parameter tuning using tree growth algorithm (TGA). As previously stated, convolution models can work on a single image and transform it from input pixel to matrix/vector representation. Current CNN pretrained models are used for feature extraction. The main goal is that CNN may not be trained, but training may be provided by the BP errors from the LSTM-DL classifiers via CNN multiple input images. Convolutional neural networks (CNNs) are used because of their improved transferability. Knowledge of this cutting-edge technology will benefit not just researchers who use CNN for radiology and medical imaging jobs but also clinical radiologists, since deep learning may influence their practise in the near future. Following CNN training, medical professionals or computer-aided detection (CADe) systems can specify the target lesions in medical pictures during the deployment phase.  Figure 2 depicts a general LSTM cell. The LSTM cell contains various gates and parameters that control the behaviour of each memory cell. Every cell state is governed by the activation function of gates. For different types of gates, the input value is fed into the input gate (I), forget gate (f), activation vector (c), and output gate (o).

(12) $$\begin{array}{c} j_{t}=\in j\left(w_{pj}p_{t}+w_{hj}h_{t-1}+w_{aj}a_{t-1}+bj\right),\\ f_{t}=\in f\left(wPp_{t}+w_{h}h_{t-1}+w_{af}a_{-1}+bf\right),\\ a_{t}=f_{t}a_{t-1}+j_{t}\in_{a}\left(w_{pc}p_{t}+w_{ha}h_{t-1}+ba\right),\\ 0_{t}=\in_{o}\left(w_{po}p_{t}+w_{hot-1}h+w_{ao}a_{t-1}+bo\right),\\ h_{t}=0_{t}\in h\left(a_{t}\right), \end{array}$$

where *w*_*pj*_, *w*_*hj*_, *w*_*aj*_, *w*_*hf*_, *w*_*af*_, *w*_*pa*_, *w*_*ha*_, *w*_*po*_, and *w*_*ao*_ denote weight (input weight, hidden weight, output weight, etc.) and *b*_*j*_, *b*_*f*_, *b*_*a*_, and *b*_0_ indicate the bias weight [21].

Each time step includes a single CNN series and an LSTM model. As a single step, CNN could be passed and used on every output to the LSTM input image for all input images. The result could be achieved by folding up a CNN input framework with multiple layers in a time distribution method. The same layer is used multiple times to achieve a similar result. To determine the presence of diseases, the extracted features are fed into the ELM classifier. Assume a training data *A*{(*x*_*i*_, *t*_*i*_)}_*i*=1_^*N*^, the output functions of SLFN using *L* hidden neuron could be determined by

(13) $$\begin{array}{c} f\left(x_{i}\right)=\sum_{j=1}^{L}\beta_{j}h_{j}\left(a_{j},b_{j},x_{i}\right)=h\left(x_{i}\right)\beta ,i=1,\ldots ,N, \end{array}$$

where *β*=*β*_1_,…, *β*_*L*_^*T*^ denotes the output weight matrix and *h*(*x*_*i*_)=[*h*_1_(*a*_1_, *b*_1_, *x*_*i*_),…, *h*_*j*_(*a*_*L*_, *b*_*L*_, *x*_*i*_)] represents the network output equivalent to the training samples *x*_*i*_.*h*_*j*_(·) indicates a nonlinear piecewise continuous function and *a*_*j*_ ∈ *R*^*d*^, and *b*_*j*_ ∈ *R*(*j*=1,2,…, *L*) means a parameter of *j*th hidden node. The training network is to discover appropriate network parameters for minimizing the error functions ‖*Hβ* − *T*‖_2_, where

(14) $$\begin{array}{c} H=\left[\begin{array}{c} h\left(x_{1}\right)\\ \vdots \\ h\left(x_{N}\right) \end{array}\right],\\ T=\left[\begin{array}{c} t_{1}^{T}\\ \vdots \\ t_{N}^{T} \end{array}\right]. \end{array}$$

It represents an SLFN using an *L* hidden neuron and denotes the hidden, output matrix, and target output.

ELM uses arbitrary hidden node parameters and the tune-free trained approach to FFNN instead of iteratively upgrading network parameters as in traditional gradient descent algorithms. ELM is flexible because it employs a hidden activation function, as demonstrated by the universal approximate ability theorem. Almost any nonlinear piecewise continuous function and its linear combination perform well in the ELM algorithm [22]. The extreme learning machine (ELM) is a fast convergent training method for single hidden layer feedforward neural networks (SLFNs). This type of SLFN allows for faster convergence training and avoids the need for many iterations to update the hidden layer weights. Compared to other classical learning algorithms in applications with increasing noise, ELM appears to outperform ELM in regression and classification tests. With a single hidden layer of neurons and random feature mapping, an ELM model learns quicker than other models. High dimensions and large data sets have aroused substantial scholarly interest in the low computing complexity.

The TGA is used to optimise the ELM model's parameter computation, resulting in improved overall classification performance. The TGA approach is stimulated by the competition between trees in the forest. A tree's attention is divided between food and sunlight. Exploration and exploitation are the two major stages of the approach. During the exploration stage, the tree moves toward the sunlight, allowing it to investigate new locations. The tree is now fulfilled with light in the exploitation stage, and thus, it moves towards better nutrients in the root, as it moves towards the global/local optimal. The forest's tree population is classified into four types.

The first group of trees has found a light source, and they can now compete for food. To compete with light, the tree in the second group switches to the two optimal options that are closest to it. In the third group, a new tree is planted in place of the worst tree. Finally, an optimal tree is used to create a novel plant [23]. Initially, this approach arbitrarily creates the early population of the tree (solution) within the lower and upper bounds, where the fitness values for all solutions are calculated. The following is how the early population is produced.

(15) $$\begin{array}{c} x_{i,j}={\text{min}}_{j}+\text{rand}\cdot \left({\text{max}}_{j}-{\text{min}}_{j}\right), \end{array}$$

where *x*_*i*,*j*_ is the *j*th variable of *i*th solution of the population, rand represents an arbitrary value derived by the uniform distribution, and min_*j*_ and max_*j*_ indicates lower bound and upper bound of *j*th variable, respectively.

Next, the population is arranged based on the fitness values, and the present optimal solution at the *j*th iterations is established. The global optimal solutions are represented as *T*_*GB*_^*j*^. The optimal solution is allocated to the initial group (*N*_1_), and the solution from this population carries out the local search as follows:

(16) $$\begin{array}{c} T_{i}^{j+1}=\frac{T_{i}^{j}}{\theta }+r\times T_{i}^{j}, \end{array}$$

where *T*_*i*_^*j*+1^ represents the novel *i*th solution and *T*_*i*_^*j*^ is the *i*th solution in *j*th iteration. *θ* represents the rate of power decreases, and *r* specifies an arbitrary number between [0,1].

When the novel solution has a higher fitness value than the current solution, greedy selections are used to find it. The novel solution either replaces the current one or keeps the current solutions for the next generation.

The second optimal solution is allocated to *N*_2_ subpopulation. All solutions from the *N*_2_ group must be shifted to the two nearest solutions (from the initial and second subpopulation) at distinct *α* angles. The Euclidean distance is used to measure the distance between two solutions.

(17) $$\begin{array}{c} d_{i}={\left(\sum_{i=1}^{N_{1}+N_{2}}{\left(T_{N_{2}}^{j}-T_{i}^{j}\right)}^{2}\right)}^{1/2},\\ d_{i}=\left\{\begin{array}{c} d_{i}\text{ if}T_{N_{2}}^{j}\neq T_{i}^{j},\\ \infty \text{ if}T_{N_{2}}^{j}=T_{i}^{j}, \end{array}\right. \end{array}$$

where *d*_*j*_ denotes the distance of *i*th solution, The trees that exist now are depicted as *T*_*N*_2__^*j*^, and the *i*th solution in the population are signified as *T*_*i*_^*j*^.

The poorest solution from the population is found in the third subpopulation, *N*_3_. This solution is calculated by replacing it with a recent arbitrary solution.

(18) $$\begin{array}{c} N_{3}=N-N_{1}-N_{2}, \end{array}$$

where the population sizes are represented by *N*.*N*_1_ and *N*_2_ are the first and second subpopulation, respectively. Next, the novel population (*N*) is determined by adding the initial groups *N*_1_, *N*_2_, and *N*_3_.

(19) $$\begin{array}{c} N=N_{1}+N_{2}+N_{3}. \end{array}$$

The last group *N*_4_ includes arbitrary novel results.*N*_4_ is the final group of entire set outcomes which contains arbitrary novel findings.. Using mask operators, the population adapts an optimal solution from the initial group (*N*), and the adapted solution is fused. The fitness values are used to organise the novel population, and the best *N* solution is chosen for the next iteration. The procedure is repeated until the desired result is obtained. Finally, the best solution is determined.

## 4. Performance Validation

The performance of the MR-LSDGM approach is investigated in this section using the benchmark activity recognition data set from the UCI repository [24]. The data set contains information on 30 people, each with 561 attributes. The data set contains 496 instances from the Walk class, 471 instances from the Up class, 420 instances from the Down class, 491 instances from the Sitting class, 532 instances from the Standing class, and 537 instances from the Lying class.

After five repetitions, the MR-LSDGM approach produced a collection of five confusion matrices, as shown in Figure 3. The graph shows that the MR-LSDGM method yielded the best possible result in each execution run [25]. For example, the MR-LSDGM technique classified 493 instances as Walk, 464 instances as Up, 415 instances as Down, 447 instances as Sit, 506 instances as Stand, and 537 instances as Lay under run-1. Similarly, the MR-LSDGM approach classified 495 instances as Walk, 466 instances as Up, 416 instances as Down, 451 instances as Sit, 510 instances as Stand, and 537 instances as Lay in run-2. Similarly, the MR-LSDGM method classified 495 instances as Walk, 464 instances as Up, 416 instances as Down, 450 instances as Sit, 508 instances as Stand, and 536 instances as Lay under run-4. Furthermore, under run-5, the MR-LSDGM algorithm classified 495 instances as Walk, 464 instances as Up, 415 instances as Down, 453, Sit, 506, Stand, and 534 instances as Lay [26].

The classification result analysis of the MR-LSDGM technique under varying execution runs is reported in Table 1 and Figure 4. The MR-LSDGM technique has resulted in superior performance across all runs, as shown in Table 1. For example, the MR-LSDGM technique achieved maximum performance with run-1, with an average sensitivity of 0.971, specificity of 0.994, precision of 0.972, accuracy of 0.990, and *F*-score of 0.972. The MR-LSDGM method also performed optimally in run-2, with an average sensitivity of 0.976, specificity of 0.995, precision of 0.977, accuracy of 0.992, and *F*-score of 0.976. Furthermore, with run-3, the MR-LSDGM method achieved an average sensitivity of 0.973, specificity of 0.994, precision of 0.973, accuracy of 0.991, and *F*-score of 0.973. With run-5, the MR-LSDGM approach improved efficiency, achieving an average sensitivity of 0.973, specificity of 0.995, precision of 0.974, accuracy of 0.991, and *F*-score of 0.973.

Figure 5 depicts the ROC analysis of the MR-LSDGM method on the applied data set under various runs [27]. According to the results, the MR-LSDGM approach had the highest ROC value in every run. For example, in run-1, the MR-LSDGM technique achieved an increased ROC of 99.9888. In line with run-2, the MR-LSDGM method has a better ROC of 99.7676. The MR-LSDGM methodology then achieved a maximum ROC of 99.9874 in run-3. Concurrently, the MR-LSDGM technique achieved a superior ROC of 99.9721 in run-4. Finally, under run-5, the MR-LSDGM method achieved a maximum ROC of 99.9416 [28].

An extended comparison analysis is provided in Table 2 [25] to demonstrate the improved performance of the MR-LSDGM technique. With accuracy of 0.9375 and 0.9531, respectively, the CNN-2016 and CC-2018 approaches produced ineffective results [29]. At the same time, the CNN-LSTM and lightweight CNN approaches improved their accuracy to 0.9627 and 0.958, respectively. Furthermore, the CNN-BiLSTM and CNN-SF approaches have acceptable accuracy values of 0.9705 and 0.9763, respectively. In contrast, the proposed MR-LSDGM approach achieved an effective performance of 0.991 [30].

As evidenced by the tables and statistics above, the MR-LSDGM technique is clearly more effective than the other procedures.

### 4.1. Discussion

The healthcare IoT data sets and performance criteria for the proposed MR-LSGDM strategy are briefly outlined in this section [31]. The complete approach was developed using the MATLAB 2021a tool on a Core i3-3110M processor running Windows 8 with 2 GB RAM, and it was tested on 8 healthcare IoT data sets (Table 1) [32]. Over 30 separate runs, the new BBO-FCM approach was compared to existing algorithms such as CNN 2016, CNN 2018, CNN-SF, CNN-LSTM, lightweight CNN, and CNN-BiLSTM in terms of intracluster distance, purity index, standard deviation, root mean square error, accuracy, and *F*-measure [33].

## 5. Conclusion

The MapReduce tool is used in this study to create a new MR-LSDGM approach for the healthcare sector. The MR-LSDGM approach includes BBO-FCM-based DM clustering, 2TFLR-based preference modelling, and LSTM-OELM-based classification procedures. To manage big data in the healthcare sector, the MR-LSDGM technique employs the MapReduce tool. Furthermore, the design of the BBO algorithm for determining the primary cluster centres of the FCM technique, as well as parameter optimization of ELM using the TGA technique, contribute to improved overall classification results. A large number of simulations are run to demonstrate the improved outcomes of the MR-LSDGM technique, and the experimental results are examined using several metrics. According to the simulation results, the MR-LSDGM methodology outperformed the other methods. In the future, the model presented here could be used in telemedicine applications to help patients in remote areas.

## Figures and Tables

**Figure 1:** Overall process of MR-LSDGM model.

**Figure 2:** LSTM structure.

**Figure 3:** Confusion matrix analysis of MR-LSDGM model.

**Figure 4:** Result analysis of MR-LSDGM model with different measures.

**Figure 5:** ROC analysis of MR-LSDGM model.

**Table 1:** Result analysis of MR-LSDGM technique under different runs.

No. of runs	Methods	Sensitivity	Specificity	Precision	Accuracy	*F*-score
Run-1	Walk	0.994	1.000	1.000	0.999	0.997
	Up	0.985	0.997	0.985	0.995	0.985
	Down	0.988	0.998	0.986	0.996	0.987
	Sit	0.910	0.989	0.943	0.976	0.926
	Std	0.951	0.981	0.918	0.976	0.934
	Lay	1.000	1.000	1.000	1.000	1.000
	**Average**	**0.971**	**0.994**	**0.972**	**0.990**	**0.972**

Run-2	Walk	0.998	1.000	1.000	1.000	0.999
	Up	0.989	0.998	0.992	0.997	0.990
	Down	0.991	0.998	0.991	0.997	0.991
	Sit	0.919	0.991	0.952	0.979	0.935
	Std	0.959	0.983	0.926	0.979	0.942
	Lay	1.000	1.000	1.000	1.000	1.000
	**Average**	**0.976**	**0.995**	**0.977**	**0.992**	**0.976**

Run-3	Walk	0.998	1.000	1.000	1.000	0.999
	Up	0.983	0.998	0.991	0.996	0.987
	Down	0.991	0.998	0.986	0.997	0.988
	Sit	0.915	0.989	0.943	0.977	0.929
	Std	0.953	0.981	0.919	0.976	0.935
	Lay	0.996	1.000	1.000	0.999	0.998
	**Average**	**0.973**	**0.994**	**0.973**	**0.991**	**0.973**

Run-4	Walk	0.998	1.000	1.000	1.000	0.999
	Up	0.985	0.998	0.992	0.996	0.988
	Down	0.991	0.998	0.988	0.997	0.989
	Sit	0.917	0.989	0.945	0.977	0.931
	Std	0.955	0.982	0.922	0.977	0.938
	Lay	0.998	1.000	1.000	1.000	0.999
	**Average**	**0.974**	**0.995**	**0.975**	**0.991**	**0.974**

Run-5	Walk	0.998	1.000	1.000	1.000	0.999
	Up	0.985	0.998	0.989	0.996	0.987
	Down	0.988	0.998	0.988	0.997	0.988
	Sit	0.923	0.989	0.942	0.978	0.932
	Std	0.951	0.983	0.923	0.977	0.937
	Lay	0.994	1.000	1.000	0.999	0.997
	**Average**	**0.973**	**0.995**	**0.974**	**0.991**	**0.973**

**Table 2:** Comparative accuracy analysis of MR-LSDGM with other techniques.

Methods	Accuracy	Precision	ROC
CNN-2016	0.9375	0.9554	0.9454
CNN-2018	0.9531	0.9638	0.9538
CNN-SF	0.9763	0.9655	0.9555
CNN-LSTM	0.9580	0.9755	0.9655
Lightweight CNN	0.9627	0.9822	0.9722
CNN-BiLSTM	0.9705	0.9852	0.9752
MR-LSDGM	0.9910	0.9925	0.9825

## Data Availability

The manuscript contains all of the data.
